The article "Effects of Ulinastatin on Proliferation and Apoptosis of Breast Cancer Cells by Inhibiting the ERK Signaling Pathway" was retracted in 2024. Reasons: signs of a paper mill; compromised peer review; unreliable results or conclusions.

# Effects of Ulinastatin on Proliferation and Apoptosis of Breast Cancer Cells by Inhibiting the ERK Signaling Pathway

**DOI:** 10.1155/2021/9999268

**Published:** 2021-07-30

**Authors:** Zeyu Xing, Xin Wang, Jiaqi Liu, Gang Liu, Menglu Zhang, Kexin Feng, Xiang Wang

**Affiliations:** Department of Breast Cancer, National Cancer Center/National Clinical Research Center for Cancer/Cancer Hospital, Chinese Academy of Medical Sciences and Peking Union Medical College, Beijing 10021, China

## Abstract

**Purpose:**

To explore the effects of ulinastatin on the proliferation and apoptosis of breast cancer cells and the relevant mechanism of action.

**Methods:**

Breast cancer cells (MCF-7) were cultured and randomly divided into three groups, namely, control group, ulinastatin group, and ulinastatin+extracellular-regulated protein kinase (ERK) inhibitor group. Then, the Cell Counting Kit-8 (CCK-8) assay was carried out to detect the effect of ulinastatin on the viability of breast cancer cells. The effects of ulinastatin on the proliferation and apoptosis of breast cancer cells were determined via EdU staining and Hoechst 33258 staining assays, respectively. The messenger ribonucleic acid (mRNA) and protein expression levels of ERK and forkhead box O3 (FOXO3) in breast cancer cells were measured through reverse transcription-polymerase chain reaction (RT-PCR) and Western blotting.

**Results:**

In comparison with the control group, the ulinastatin group displayed decreased viability of breast cancer cells, a decreased positive rate of 5-ethynyl-2′-deoxyuridine (EdU) staining, an increased positive rate of Hoechst 33258 staining, and reduced mRNA and protein levels of ERK and FOXO3 in breast cancer cells. Compared with those in the ulinastatin group, the viability of breast cancer cells was lowered, the positive rate of EdU staining was reduced, the positive rate of Hoechst 33258 staining was raised, and the mRNA and protein levels of ERK and FOXO3 in breast cancer cells clearly declined in the ulinastatin+ERK inhibitor group.

**Conclusion:**

Ulinastatin inhibits the proliferation and promotes the apoptosis of breast cancer cells. The possible mechanism of action is associated with the suppression of the ERK signaling pathway.

## 1. Introduction

Breast cancer, one of the most common malignancies among women in China and even in the world at present, has become the leading killer threatening the health of women, which accounts for about 20% of malignant tumors among women [1]. With the deepening of studies, it is found by researchers that patients with breast cancer are younger in recent years, and the incidence rate of breast cancer is increasing year by year with enhanced social survival and work stress [2, 3]. Reports of the World Health Organization have stated that about 1.5 million people suffer from breast cancer every year worldwide, and about 500,000 patients with breast cancer die. With continuous improvement and perfection of modern medicine, certain progress has been made in the prevention and treatment of breast cancer, mainly including chemoradiotherapy, surgery, or endocrine therapy [4]. Recently, medical practitioners apply some targeted inhibitors in clinical treatment, but the efficacy is unsatisfactory. Therefore, further investigating the pathogenesis of breast cancer and finding out drugs preventing or treating breast cancer are major issues to be solved.

The article "Effects of Ulinastatin on Proliferation and Apoptosis of Breast Cancer Cells by Inhibiting the ERK Signaling Pathway" was retracted in 2024. Reasons: signs of a paper mill; compromised peer review; unreliable results or conclusions.

In recent years, a large amount of literature evidence has manifested that the mitogen-activated protein kinase (MAPK) signaling pathway plays a crucial role in the proliferation, differentiation, and apoptosis of cells [5]. As one of the most important signal transduction pathways in the MAPK signaling pathway, the extracellular-regulated protein kinase (ERK) signaling pathway has abnormal changes in the case of breast cancer [6]. ERK cascade reaction can be stimulated by various signals like tyrosine kinase and G protein-coupled receptor signal, which participates in the modulation of many processes including the proliferation, apoptosis, and invasion of breast cancer cells. Forkhead box O3 (FOXO3), a downstream target of ERK, is regulated by ERK [7]. FOXO3 belongs to FOXO, whose abnormal expression may be closely correlated with the development and progression of tumors [8]. Repressing the ERK signaling pathway may be a new way to treat breast cancer.

Ulinastatin (molecular formula: C13H16O3) is a urinary trypsin inhibitor (UTI) and a glycoprotein containing 143 amino acids, chemically named 3-(furan-2-yl)-2,4-dioxaspiro [5.5] undec-9-ene and mainly applied in the treatment of acute pancreatitis or chronic recurrent pancreatitis in clinical practice [9]. Recent studies have found that ulinastatin has an outstanding effect in inhibiting tumor progression and can notably inhibit the proliferation, migration, and invasion of lung cancer cells [10]. Moreover, Song et al. discovered that ulinastatin suppresses the proliferation of live cancer cells, and the mechanism may be related to the inhibition of autophagy [11]. Zhao et al. revealed that ulinastatin inhibits the growth of breast cancer cells and the expressions of interleukin-6, interleukin-8, and tumor necrosis factor-*α* [12]. The above research results suggest that ulinastatin plays an important role in modulating the development and progression of tumors. However, the mechanism by which ulinastatin regulates the proliferation and apoptosis of breast cancer cells remains unclear and needs to be further studied.

The article "Effects of Ulinastatin on Proliferation and Apoptosis of Breast Cancer Cells by Inhibiting the ERK Signaling Pathway" was retracted in 2024. Reasons: signs of a paper mill; compromised peer review; unreliable results or conclusions.

## 2. Reagents, Instruments, and Cells

### 2.1. Reagents

The following were purchased from their respective manufacturers: P/S, fetal bovine serum (FBS), and Dulbecco's modified Eagle medium- (DMEM-) H medium (Gibco, USA), Cell Counting Kit-8 (CCK-8) (GlpBio, USA), 96-well culture plates and culture dishes (Corning, USA), 5-ethynyl-2′-deoxyuridine (EdU) staining solution (Sigma, USA), Hoechst 33258 staining solution (Solarbio, Beijing), ERK and FOXO3 primers (Thermo Fisher, USA), ERK and FOXO3 primary antibodies (Shenyang Wanlei Biotechnology Co., Ltd.), fluorescein isothiocyanate- (FITC-) labeled IgG secondary antibody (Jackson, USA), and first-strand complementary deoxyribonucleic acid (cDNA) synthesis kit (Hangzhou Xinjing Bio-Agent Development Co., Ltd.).

### 2.2. Instruments

A microplate reader (bought from Beijing Perlong New Technology Co., Ltd.), a CO_2_ incubator (Contherm, New Zealand), a polymerase chain reaction (PCR) instrument and an electrophoresis instrument (Bio-Rad, USA), a gel imager (LongGene Instruments, Hangzhou), and a membrane scanner (Thermo Fisher, USA) were used.

### 2.3. Cells

Human breast cancer cells (MCF7) used in this study were purchased from Shanghai Yaji Biotechnology Co., Ltd. Complete medium included 1% P/S, 10% FBS, and DMEM-H medium. The breast cancer cells were randomly divided into the control group, ulinastatin group (800 U/mL), and ulinastatin+ERK inhibitor group (800 U/mL+500 nM).

## 3. Methods

### 3.1. Detection of Effect of Ulinastatin on the Viability of Breast Cancer Cells via the CCK-8 Assay

Cell suspension (100 *μ*L) was inoculated into a 96-well plate, with three replicate wells set for each group, and cultured in the 5% CO_2_ incubator overnight. 800 U/mL ulinastatin was given in the ulinastatin group, while 800 U/mL ulinastatin and 500 nM ERK inhibitor solution were given in the ulinastatin+ERK inhibitor group. After that, the cell viability was examined at 24 h, 48 h, and 72 h, respectively, and CCK-8 (10 *μ*L) was added to each well for culture for 4 h. Lastly, the absorbance was measured at 450 nm using the microplate reader.

### 3.2. Determination of Effect of Ulinastatin on the Proliferation of Breast Cancer Cells through the EdU Staining Assay

EdU, a thymidine nucleoside analogue, can be inserted into a DNA molecule being replicated during cell proliferation, which is used to detect the proliferation of cells. The cells in each group were fixed, permeabilized with 0.05% Triton X-100 solution for 15 min, added with EdU working solution, and incubated in a dark place for 30 min. After that, the working solution was washed with phosphate-buffered saline (PBS) solution, and the cells were added with an antifluorescence quencher. Lastly, a fluorescence microscope was used to observe the staining.

The article "Effects of Ulinastatin on Proliferation and Apoptosis of Breast Cancer Cells by Inhibiting the ERK Signaling Pathway" was retracted in 2024. Reasons: signs of a paper mill; compromised peer review; unreliable results or conclusions.

### 3.3. Detection of Effect of Ulinastatin on Apoptosis of Breast Cancer Cells by the Hoechst 33258 Staining Assay

Hoechst 33258 is a kind of blue fluorescent dye that can penetrate cell membranes, which is almost nontoxic to cells. In the case of apoptosis, the nucleus of apoptotic cells is fragmented and pyknotic after Hoechst 33258 staining, so that Hoechst 33258 is often used to detect apoptosis. After fixation, each group of cells was washed with PBS, added dropwise with Hoechst 33258 staining solution diluted with PBS solution at 1 : 100, incubated for 5 min, and washed with PBS for 3 times (5 min/time), followed by observation of the staining directly using the fluorescence microscope.

### 3.4. Determination of Effect of Ulinastatin on Messenger Ribonucleic Acid (mRNA) Levels of ERK and FOXO3 in Breast Cancer Cells by Means of Reverse Transcription- (RT-) PCR

Breast cancer cells in each group were taken, and total RNAs were extracted using TRIzol lysis buffer and diluted until the concentration reached 1 *μ*g/*μ*L. The cDNA was synthesized according to the instructions, and 4 *μ*L of 5× RT buffer, 2 *μ*L of RT enzyme mix buffer, and 4 *μ*L of RT primer mix buffer were sequentially added, heated at 42°C for 15 min, incubated at 95°C for 3 min, and placed on ice. Then, PCR amplification was carried out for a total of 35 cycles. 1 *μ*L of forward (F) and 1 *μ*L of reverse (R) primers were added. The primer information is shown in Table 1. The product after the amplification was subjected to gel electrophoresis. The statistics of PCR bands was conducted using ImageJ software.

### 3.5. Detection of Effect of Ulinastatin on Protein Expression Levels of ERK and FOXO3 in Breast Cancer Cells with the Help of Western Blotting

Total protein was extracted from each group of cells with the RIPA reagent, and the concentration of total protein in each group was determined by the BCA assay. Total protein samples (30 *μ*g) were loaded and separated by 10% SDS-PAGE. After that, a wet membrane transfer box (Bio-Rad) was employed to transfer the protein to a PVDF membrane, and then, the membrane was blocked with 5% skim milk powder solution for 1 h and incubated with PI3K and AKT primary antibodies overnight, washed with TBST solution for 5 min for 3 times, and incubated with an FITC-labeled secondary antibody for 1 h. Lastly, band images were obtained on the membrane scanner.

### 3.6. Statistical Analysis

All assays were repeated for at least 3 times. SPSS 18.0 analysis software was utilized to analyze and calculate data, and the results were expressed as mean ± standard deviation. Analysis of variance was applied for the significance of difference, and *p* < 0.05 suggested that the difference was statistically significant.

The article "Effects of Ulinastatin on Proliferation and Apoptosis of Breast Cancer Cells by Inhibiting the ERK Signaling Pathway" was retracted in 2024. Reasons: signs of a paper mill; compromised peer review; unreliable results or conclusions.

## 4. Results

### 4.1. Ulinastatin Inhibited the Viability of Breast Cancer Cells

The results of the CCK-8 assay shown in Figure 1 revealed that compared with that in the control group, the viability of breast cancer cells decreased significantly in the ulinastatin group at 24 h, 48 h, and 72 h (^∗^*p* < 0.05, ^∗^*p* < 0.05, and ^∗^*p* < 0.05), while it was overtly lower in the ulinastatin+ERK inhibitor group than in the ulinastatin group (^#^*p* < 0.05, ^#^*p* < 0.05, and ^#^*p* < 0.05), indicating that ulinastatin represses the viability of breast cancer cells, and the inhibitory effect is more obvious after using the ERK inhibitor.

### 4.2. Ulinastatin Suppressed Proliferation of Breast Cancer Cells

The results of EdU staining are shown in Figure 2(a). The proliferation rate of breast cancer cells was evidently reduced in the ulinastatin group compared with the control group (^∗^*p* < 0.05), and it declined in the ulinastatin+ERK inhibitor group compared with the ulinastatin group (^#^*p* < 0.05), implying that ulinastatin inhibits the proliferation of breast cancer cells, and the inhibitory effect is more evident after the use of the ERK inhibitor.

### 4.3. Ulinastatin Promoted Apoptosis of Breast Cancer Cells

The results of Hoechst 33258 staining shown in Figure 3(a) showed that apoptotic cells were shrunk and fluorescent. The apoptosis rate of breast cancer cells was higher in the ulinastatin group than in the control group (^∗^*p* < 0.05), and it was raised in the ulinastatin+ERK inhibitor group compared with the ulinastatin group (^#^*p* < 0.05), suggesting that ulinastatin can facilitate the apoptosis of breast cancer cells, and apoptosis is more remarkable after using the ERK inhibitor.

### 4.4. Ulinastatin Inhibited mRNA Levels of ERK and FOXO3 in Breast Cancer Cells

According to RT-PCR bands shown in Figure 4(a), the ulinastatin group had markedly decreased mRNA levels of ERK and FOXO3 in breast cancer cells compared with the control group (^∗^*p* < 0.05, ^∗^*p* < 0.05), and the ulinastatin+ERK inhibitor group exhibited obviously reduced mRNA levels of ERK and FOXO3 in breast cancer cells compared with the ulinastatin group (^#^*p* < 0.05, ^#^*p* < 0.05), indicating that ulinastatin is capable of repressing the mRNA expressions of ERK and FOXO3 in the ERK signaling pathway.

### 4.5. Ulinastatin Suppressed Protein Levels of ERK and FOXO3 in Breast Cancer Cells

Western blotting bands shown in Figure 5(a) revealed that the protein levels of ERK and FOXO3 in breast cancer cells were notably lower in the ulinastatin group than in the control group (^∗^*p* < 0.05, ^∗^*p* < 0.05), and they were also remarkably lower in the ulinastatin+ERK inhibitor group than in the ulinastatin group (^#^*p* < 0.05, ^#^*p* < 0.05), suggesting that ulinastatin inhibits the protein expressions of ERK and FOXO3 in the ERK signaling pathway.

The article "Effects of Ulinastatin on Proliferation and Apoptosis of Breast Cancer Cells by Inhibiting the ERK Signaling Pathway" was retracted in 2024. Reasons: signs of a paper mill; compromised peer review; unreliable results or conclusions.

## 5. Discussion

As one of the most common cancers among women in the world, breast cancer has an increasing incidence rate year by year [13]. Its pathogenesis is closely related to personal diet, living habits, and environmental factors. In clinical practice, surgical treatment is mainly adopted to treat the disease, which is supplemented by chemotherapy, radiotherapy, or small molecular targeted therapy due to diverse biological properties of breast cancer. However, the treatment effect on patients with advanced breast cancer is unsatisfactory, and chemotherapy and radiotherapy result in adverse reactions in the body of patients, severely affecting the quality of life of patients [14]. Therefore, developing safe and effective new therapeutic drugs and improving therapeutic effect have become hot spots in the field of breast cancer research.

As a UTI, ulinastatin is mainly used to treat pancreatitis [15, 16]. In recent years, researchers have discovered that ulinastatin is very effective in inhibiting tumor development and metastasis. A study of in vitro regulation on gastric cancer SGC-7901 cells conducted by Wang et al. has pointed out that ulinastatin serves as a broad-spectrum protease UTI and is able to distinctly inhibit the proliferation and migration of gastric cancer SGC-7901 cells, implying that ulinastatin may be a potential strategy for the treatment of gastric cancer [17]. Shen et al. found that ulinastatin represses the metastasis of liver cancer cells by regulating the expressions of matrix metalloproteinase-9 and E-cadherin, and its effect is more evident when combining with curcumin [18]. More and more literatures have proven the antineoplastic effect of ulinastatin, while its regulatory effect in breast cancer is rarely reported.

Therefore, in this study, the viability of breast cancer cells in each group was firstly detected via the CCK-8 assay, and the results suggest that ulinastatin significantly inhibits the viability of breast cancer cells. Next, the effects of ulinastatin on the proliferation and apoptosis of breast cancer cells were examined. The results of EdU staining indicate that ulinastatin clearly suppresses the proliferation of breast cancer cells, and Hoechst 33258 staining results imply that ulinastatin remarkably promotes the apoptosis of breast cancer cells. Uncontrolled proliferation and undifferentiation are the most obvious features of tumor cells. The pathogenesis of breast cancer is closely associated with the unlimited proliferation of breast cancer cells. Numerous studies have demonstrated that the ERK signaling pathway is a key participant in the development and progression of breast cancer. For instance, Peng et al. found that knocking out Linc-RoR can improve the stability of DUSP7 protein and inhibit the proliferation of breast cancer cells, and the mechanism may be related to the inhibition of ERK phosphorylation [19]. Research of breast cancer tissues and adjacent tissues performed by Li et al. has revealed that the expression of AKR1B10 in breast cancer tissues is overtly increased and positively correlated with tumor size and metastasis, and the overexpression of AKR1B10 promotes the proliferation and invasion of breast cancer cells, and its mechanism may be related to the activation of the ERK signaling pathway [20]. The above results indicate that the ERK signaling pathway is an important factor in the development and progression of breast cancer. To further explore the mechanism of ulinastatin in the proliferation and apoptosis of breast cancer cells, the expressions of ERK and FOXO3, key factors in the ERK signaling pathway, were examined at the gene and protein levels in this study, and the results imply that ulinastatin markedly suppresses the expressions of ERK and FOXO3, and the effect is more significant after the use of the ERK inhibitor.

The article "Effects of Ulinastatin on Proliferation and Apoptosis of Breast Cancer Cells by Inhibiting the ERK Signaling Pathway" was retracted in 2024. Reasons: signs of a paper mill; compromised peer review; unreliable results or conclusions.

In conclusion, ulinastatin reduces the expressions of ERK and FOXO3 by inhibiting the ERK signaling pathway, thereby repressing the proliferation and promoting the apoptosis of breast cancer cells. However, whether it can exert therapeutic effects in other tumors through such a mechanism of action needs to be further explored.

## Figures and Tables

**Figure 1:** Cell viability detected by the CCK-8 assay (^∗^*p* < 0.05: ulinastatin group vs. control group, ^#^*p* < 0.05: ulinastatin+ERK inhibitor group vs. ulinastatin group).

**Figure 2:** Effect of ulinastatin on breast cancer cell proliferation: (a) picture of EdU staining (20×); (b) proliferation rate (^∗^*p* < 0.05: ulinastatin group vs. control group, ^#^*p* < 0.05: ulinastatin+ERK inhibitor group vs. ulinastatin group).

**Figure 3:** Effect of ulinastatin on apoptosis of breast cancer cells: (a) picture of Hoechst 33258 staining (20×); (b) apoptotic rate (^∗^*p* < 0.05: ulinastatin group vs. control group, ^#^*p* < 0.05: ulinastatin+ERK inhibitor group vs. ulinastatin group).

The article "Effects of Ulinastatin on Proliferation and Apoptosis of Breast Cancer Cells by Inhibiting the ERK Signaling Pathway" was retracted in 2024. Reasons: signs of a paper mill; compromised peer review; unreliable results or conclusions.

**Figure 4:** mRNA levels of ERK and FOXO3 in breast cancer cells detected via RT-PCR: (a) bands of RT-PCR; (b) analysis of the bands (^∗^*p* < 0.05: ulinastatin group vs. control group, ^#^*p* < 0.05: ulinastatin+ERK inhibitor group vs. ulinastatin group).

**Figure 5:** Protein levels of ERK and FOXO3 in breast cancer cells measured through RT-PCR: (a) bands of Western blotting; (b) analysis of the bands (^∗^*p* < 0.05: ulinastatin group vs. control group, ^#^*p* < 0.05: ulinastatin+ERK inhibitor group vs. ulinastatin group).

**Table 1:** Information of primers.

List	F primer	R primer
ERK	TACACCAACCTCTCGTACATCG	CATGTCTGAAGCGCAGTAAGATT
FOXO3	CGGACAAACGGCTCACTCT	GGACCCGCATGAATCGACTAT
*β*-Actin	GGCTGTATTCCCCTCCATCG	CCAGTTGGTAACAATGCCATGT

## Data Availability

All data are available in the article.

## References

[1] Woolston C. (2015). Breast cancer. *Nature*.

[2] Anastasiadi Z., Lianos G. D., Ignatiadou E., Harissis H. V., Mitsis M. (2017). Breast cancer in young women: an overview. *Updates in Surgery*.

[3] Baade P. (2017). Geographical variation in breast cancer outcomes. *International Journal of Environmental Research and Public Health*.

[4] Castaneda S. A., Strasser J. (2017). Updates in the treatment of breast cancer with radiotherapy. *Surgical Oncology Clinics of North America*.

[5] Gu X. D., Xu L. L., Zhao H., Gu J. Z., Xie X. H. (2017). Cantharidin suppressed breast cancer MDA-MB-231 cell growth and migration by inhibiting MAPK signaling pathway. *Brazilian Journal of Medical and Biological Research*.

[6] Sun Y., Liu W. Z., Liu T., Feng X., Yang N., Zhou H. F. (2015). Signaling pathway of MAPK/ERK in cell proliferation, differentiation, migration, senescence and apoptosis. *Journal of Receptor and Signal Transduction Research*.

[7] Sampattavanich S., Steiert B., Kramer B. A., Gyori B. M., Albeck J. G., Sorger P. K. (2018). Encoding growth factor identity in the temporal dynamics of FOXO3 under the combinatorial control of ERK and AKT kinases. *Cell Systems*.

[8] Yang W., Du W. W., Li X., Yee A. J., Yang B. B. (2016). Foxo 3 activity promoted by non-coding effects of circular RNA and Foxo 3 pseudogene in the inhibition of tumor growth and angiogenesis. *Oncogene*.

[9] Wang G., Liu Y., Zhou S. F. (2016). Effect of somatostatin, ulinastatin and gabexate on the treatment of severe acute pancreatitis. *The American Journal of the Medical Sciences*.

[10] Bao P., Zhao W., Li Y., Liu Y., Zhou Y., Liu C. (2015). Protective effect of ulinastatin in patients with non-small cell lung cancer after radiation therapy: a randomized, placebo-controlled study. *Medical Oncology*.

[11] Song B., Bian Q., Shao C. H. (2015). Ulinastatin reduces the resistance of liver cancer cells to epirubicin by inhibiting autophagy. *PLoS One*.

The article "Effects of Ulinastatin on Proliferation and Apoptosis of Breast Cancer Cells by Inhibiting the ERK Signaling Pathway" was retracted in 2024. Reasons: signs of a paper mill; compromised peer review; unreliable results or conclusions.

[12] Zhao X., Sun X., Gao F., Luo J., Sun Z. (2011). Effects of ulinastatin and docataxel on breast tumor growth and expression of IL-6, IL-8, and TNF-*α*. *Journal of Experimental & Clinical Cancer Research*.

[13] Braden A., Stankowski R., Engel J., Onitilo A. (2014). Breast cancer biomarkers: risk assessment, diagnosis, prognosis, prediction of treatment efficacy and toxicity, and recurrence. *Current Pharmaceutical Design*.

[14] Libson S., Lippman M. (2014). A review of clinical aspects of breast cancer. *International Review of Psychiatry*.

[15] Li D., Ji H., Zhao B. (2018). Therapeutic effect of ulinastatin on pulmonary fibrosis via downregulation of TGF-*β*1, TNF-*α* and NF-*κ*B. *Molecular Medicine Reports*.

[16] Atal S. S., Atal S. (2016). Ulinastatin - a newer potential therapeutic option for multiple organ dysfunction syndrome. *Journal of Basic and Clinical Physiology and Pharmacology*.

[17] Wang J., Chen X., Su L., Zhu Z., Wu W., Zhou Y. (2016). Suppressive effects on cell proliferation and motility in gastric cancer SGC-7901 cells by introducing ulinastatin in vitro. *Anti-Cancer Drugs*.

[18] Shen F., Cai W. S., Li J. L. (2014). Synergism from the combination of ulinastatin and curcumin offers greater inhibition against colorectal cancer liver metastases via modulating matrix metalloproteinase-9 and E-cadherin expression. *Oncotargets and Therapy*.

[19] Peng W. X., Huang J. G., Yang L., Gong A. H., Mo Y. Y. (2017). Linc-RoR promotes MAPK/ERK signaling and confers estrogen-independent growth of breast cancer. *Molecular Cancer*.

[20] Li J., Guo Y., Duan L. (2017). AKR1B10 promotes breast cancer cell migration and invasion via activation of ERK signaling. *Oncotarget*.

